The article "Frontal Alpha Complexity of Different Severity Depression Patients" was published in 2020. Journal: J Healthc Eng.

# Frontal Alpha Complexity of Different Severity Depression Patients

**DOI:** 10.1155/2020/8854725

**Published:** 2020-09-14

**Authors:** Lulu Zhao, Licai Yang, Baimin Li, Zhonghua Su, Chengyu Liu

**Affiliations:** ^1^School of Control Science and Engineering, Shandong University, Jinan 250061, China; ^2^The Third Hospital of Jinan, Jinan 250132, China; ^3^The Second Affiliated Hospital of Jining Medical College, Jining 272051, China; ^4^School of Instrument Science and Engineering, Southeast University, Nanjing 211189, China

## Abstract

Depression is a leading cause of disability worldwide, and objective biomarkers are required for future computer-aided diagnosis. This study aims to assess the variation of frontal alpha complexity among different severity depression patients and healthy subjects, therefore to explore the depressed neuronal activity and to suggest valid biomarkers. 69 depression patients (divided into three groups according to the disease severity) and 14 healthy subjects were employed to collect 3-channel resting Electroencephalogram signals. Sample entropy and Lempel–Ziv complexity methods were employed to evaluate the Electroencephalogram complexity among different severity depression groups and healthy group. Kruskal–Wallis rank test and group *t*-test were performed to test the difference significance among four groups and between each two groups separately. All indexes values show that depression patients have significantly increased complexity compared to healthy subjects, and furthermore, the complexity keeps increasing as the depression deepens. Sample entropy measures exhibit superiority in distinguishing mild depression from healthy group with significant difference even between nondepressive state group and healthy group. The results confirm the altered neuronal activity influenced by depression severity and suggest sample entropy and Lempel–Ziv complexity as promising biomarkers in future depression evaluation and diagnosis.

## 1. Introduction

Depression is a common mental disorder with widespread influence and destruction beyond expectation. According to the World Health Organization, depression leads to approximately 800,000 suicides every year and is a leading cause of disability worldwide [1]. However, the specific pathology is little known [2] and the underlying neural activities are still under investigation [3]. Valid and effective biomarkers could contribute to exploring the pathology and the physiological variation of depression patients. Besides, the current mental diseases including depression are mainly diagnosed according to the psychiatrist's overall evaluation without any specific indexes. Accurate biomarkers could provide objective data support to clinical depression diagnosis and to the future computer-aided diagnosis as well. Nowadays, computer-aided technology plays a monumental part in all walks of life, such as the production or manufacturing of advanced devices. The basic principles and features of computer-aided approaches could be integrated into medical domain to provide potential and interesting solutions in the field of diagnosis [4].

The article "Frontal Alpha Complexity of Different Severity Depression Patients" was published in 2020. Journal: J Healthc Eng.

Among varieties of biomarkers based on multiple electrophysiology signals, Electroencephalogram (EEG) signal is the most promising one for mental disease, as it is a direct reflection of brain bioelectric activity which provides high temporal resolution for evaluation of the brain dynamics [5]. Besides, compared with methods such as functional Magnetic Resonance Imaging and biochemical indexes, it also has advantages of being noninvasive, lower cost, acquisition convenience, and so on [6]. Therefore, there are increasing researchers interested in detecting and discriminating depression patients by employing features extracted from EEG signals, from linear methods [7–9] to nonlinear methods. However, EEG signals are complex, nonlinear, and nonstationary due to the nonlinearity of the brain activity in nature [10, 11]. Therefore, nonlinear methods show obvious advantages, as the linear methods are limited in evaluating the complex dynamical variations of depression brain. Besides, the complexity of alpha band from frontal regions has become a research hotspot in depression evaluation. Theoretically, it is suggested that frontal lesions mainly lead to mental disorders, manifested as loss of memory and attention, slow response, and decreased thinking, which are also manifestations of depression [12, 13]. In addition, multiple researchers confirmed the importance and validation of frontal alpha signal in depression recognition, such as Kalev et al. [14], Hosseinifard et al. [10], Chang et al. [15], Lee et al. [16], and so on.

Interestingly, as an index which was proposed to measure both regularity and complexity of clinical and experimental time-series data [17, 18], sample entropy (SEn) has not found wide use in depressive EEG analysis, and the existing research presented inconsistent complexity results compared with other methods. For example, higher sample entropy values were found in normal class compared with depression class by both Faust and Acharya [18, 19], while on the contrary most studies employing other nonlinear complexity measures, such as Lempel–Ziv complexity (LZC), Kolmogorov complexity, Higuchi's fractal dimension, and fractal dimension proved increased complexity in depression patients compared with healthy group [5, 20]. As a nonparametric and model-independent method, LZC does not require a long data series and thus gives more reliable results in short clinical studies [21]. Based on the above analysis, SEn and LZC were employed simultaneously in this study, to confirm the complexity variation of frontal alpha band in depressive patients, especially whether these two complexity measurements lead to different complexity variation trends in the same groups of patients and healthy people. In addition, previous studies mainly focused on the nonlinear complexity difference between depression patients and healthy subjects but seldom paid attention to the complexity variation effected by the degree of depression. In this study, different severity depression patients were selected, and the correlation between frontal alpha complexity and depression severities would also be explored.

The article "Frontal Alpha Complexity of Different Severity Depression Patients" was published in 2020. Journal: J Healthc Eng.

The aim of this study is to evaluate the frontal alpha EEG variation influenced by different depression severities by employing two different complexity algorithms. As expected, consistent increased frontal complexity is suggested by both SEn and LZC measures, and furthermore, the complexity increase rises further as the depression deepens. The results confirm the variation of neuronal activity caused by depression and suggest SEn and LZC as promising biomarkers for future computer-aided depression diagnosis.

## 2. Materials and Methods

### 2.1. Subjects

69 depression patients and 14 healthy subjects were employed in this study. All participants with depression were inpatients under normal treatment recruited from the Second Affiliated Hospital of Jining Medical College, Shandong, China. Patients were diagnosed by two experienced specialists according to ICD-10 (International Classification of Diseases, 10th Edition) and the depression degrees were evaluated according to the 17-item Hamilton Depression Rating Scale (HDRS). Then, three depression groups were consisted by different severity patients according to their HDRS scores [22]: Non-De Group (0–7 scores), including 15 patients with nondepressive state; Mil-De Group (8–17), including 34 patients with mild depression; and Con-De Group (>17), including 20 patients with confirmed depression. 14 healthy subjects without any mental disorders were recruited from Shandong University, and no medicine or tea or coffee was taken in last 24 hours before data acquisition.  Table 1 provides detailed information of all subjects.

The experiment was conducted in accordance with the Declaration of Helsinki and was approved by the Ethics Committee of the Second Affiliated Hospital of Jining Medical College. Written informed consent was given by each participant.

The article "Frontal Alpha Complexity of Different Severity Depression Patients" was published in 2020. Journal: J Healthc Eng.

### 2.2. Data Acquisition and Preprocessing

EEG signals of all subjects were recorded by a multichannel physiological acquisition system, RM6280C (Chengdu Instrument Factory, Sichuan, China). According to the discussion in introduction, the frontal alpha EEG is considered as the target signal. In view of clinical operation convenience and signal effectiveness, signals from three poles including left frontal pole (Fp1), frontal zero (Fz), and right frontal pole (Fp2) were collected, as shown in Figure 1. The patch electrodes were used in poles Fp1 and Fp2, while bridge type electrode was used in Fz with an elastic electrode cap for fixation. Single lead method was applied since the three poles positions were quite near, and both ear lobes were used as indifferent electrodes. To minimize noise interference, the bridge electrode was soaked in normal saline solution, and the skin at the poles was decreased by 75% medical alcohol. A thin layer of conductive paste was also used before the electrode's fixation. The sensitive parameter was set as 100 *μ*V, and time consistent was 0.2 s. Hardware filtering was turned off to minimize valid signal losing, while the 30 Hz digital low pass filter was employed for better visual observation of signals.

Data collection procedures and matters needing attention were introduced to each subject when they entered the collection room. Depression patients were accompanied by their familiar doctor to avoid extra nerves to the strange environment. At least 5.5 min stable EEG signals were collected in supine position with eyes closed. Subjects were asked to keep the whole body relaxed and breath evenly without any movements. For more detailed collection information, one could refer to our previous article [23].

The raw EEG signals were firstly resampled from 1000 Hz to 200 Hz, and wavelet threshold filter was used to remove artifacts caused by electrooculogram. Butterworth filter was used to extract the alpha band signal (8–13 Hz). Then, each signal was checked visually to remove the abnormal data segment, such as extremely high or low points which were beyond the scope of mean ± triplicate standard deviation, or the long zero series which might happen when valid signal was covered by strong noise. Finally, 5 min clear alpha EEG was kept for the following feature extraction.

### 2.3. Feature Extraction

Entropy-based measures, such as approximate entropy and SEn, as nonlinear measurements to value the regularity of short physiological time series, have been widely used to explore their inherent complexity [24]. SEn is an improved entropy measure because it overcomes the biased estimation problem that happens in approximate entropy caused by self-matches [15]. SEn estimates the signal complexity by calculating the conditional probability that two series of a given length *n*, similar for *m* points, remain similar within tolerance *r* at the next data point. A higher SEn value suggests a lower regularity and increased complexity of the time series. According to a previous study [25], embedding dimension *m* of 2 and 3 and tolerance threshold *r* of 0.10 and 0.15 were recommended by Zhao et al. Different combinations of the above suggested parameters were compared, and finally *m* = 2 and *r* = 0.1 were employed.

The article "Frontal Alpha Complexity of Different Severity Depression Patients" was published in 2020. Journal: J Healthc Eng.

LZC was proposed by Lempel and Ziv [26] to evaluate the complexity of a finite length series. Different from entropy measures, LZC values the sequence complexity by counting the rate of new patterns appearing in a time series. According to the definition of LZC, the series should be a binary sequence firstly. Previous studies have proved that taking the median value of the time series as the binary threshold is more robust to outliers [27]. Then, the resulting binary sequence was scanned from left to right to count the number of new patterns. For detailed calculation of LZC, please refer to [28].

### 2.4. Statistical Analysis

The whole process of data preprocessing, feature extraction, and statistical analysis was performed in MATLAB (Ver. R2019a, MathWorks, United States). Normal distribution was tested firstly, and for the parameters which passed the test, one-way ANOVA and group *t*-test were employed to test the difference among all four groups and the difference between each two groups separately. Otherwise, for parameters which failed the normal distribution test, the Kruskal–Wallis rank test and Wilcoxon rank sum test were performed instead. Besides, the correlations between HDRS scores and index values were explored by Pearson correlation analysis. Healthy group was not included in the correlation analysis as there were no HDRS scores for them. Statistical significance with *p* value lower than 0.05 was admitted for all statistical results.

## 3. Results

The overall results confirmed discriminability of both SEn and LZC employed in this study among different groups, especially between depression and healthy groups, which indicated altered frontal complexity in depression patients.

### 3.1. Difference Analysis

According to the above feature extraction and statistical analysis, 6 indexes were acquired finally for each group: SEn measures of three channels, which are SEn_Fp1, SEn_Fz, and SEn_Fp2; LZC measures of three channels, which are LZC_Fp1, LZC_Fz, and LZC_Fp2.

There is no index among the four groups that passed the normal distribution and variance homogeneity test both; therefore, the Kruskal–Wallis rank test was used instead of the one-way ANOVA. The difference results are shown in the first two columns of Table 2. Significant difference among different depression severities and healthy subjects was confirmed for all the 6 indexes with *p* < 0.01.

The article "Frontal Alpha Complexity of Different Severity Depression Patients" was published in 2020. Journal: J Healthc Eng.

To further explore the difference between each two groups, group *t*-test was performed as follows. Among all 6 indexes of four groups, there are 12 that are of abnormal distribution; therefore, each pair of groups related to these ones was tested by Wilcoxon rank sum test. Others were analyzed by the group *t*-test. The feature values of each group are shown in the form of mean ± standard error in Table 2, and the difference significance between each pair of groups is also listed in detail.

In the complexity comparison, all entropy measures of the healthy group show significant lower values than three depression groups, whether taking different severities of depression into consideration, or in view of signal channels collected from different pole positions. It is worth highlighting that, when compared with healthy group, the entropy values of depression groups have all increased significantly with *p* < 0.01. Unfortunately, the differences are not significant enough in the comparison within depression groups, especially between the Non-De group and the other two depression groups, with only one exception; for the SEn_Fp1, it has decreased by 0.0034 from Non-De group to Mil-De group, with *p* < 0.05. However, in the comparison between Mil-De and Con-De group, two entropy measures have significant differences, with only SEn_Fz as an exception. In the case of LZC measures, there is no significant difference either between group healthy and Non-De or between Mid-De and Con-De. However, significant increases do exist in the other four group pairs, and especially all with *p* < 0.01. For better visual observation, Figure 2 shows the 6 feature values' distribution among the four groups. A general increasing trend could be perceived from these bar graphs among four groups. Curiously, a decrease happens in the Con-De group for four of the six features, with exception of LZC_Fz and LZC_Fp2.

### 3.2. Correlation Analysis

The correlation results between complexity values and HDRS values are presented in this part, as shown in Table 3 and Figure 3. Interestingly, SEn and LZC measures show up an opposite complexity changing trend. Three sample entropy values suggest negative relationships with HDRS, with −0.1284, −0.0364, and −0.0990 *R* values, and only SEn_Fp1 has significance with *p* < 0.01, and SEn_Fp2 has significance with *p* < 0.05, while there is no significant correlation for SEn_Fz. On the other hand, LZC values suggest positive relationships with HDRS, with 0.0548, 0.1067, and 0.0735 *R* values, and only LZC_Fz shows correlation significance with *p* < 0.01. However, all correlation coefficient values are quite small, which suggests a weak correlation between HDRS scores and the above feature values.

The article "Frontal Alpha Complexity of Different Severity Depression Patients" was published in 2020. Journal: J Healthc Eng.

## 4. Discussion

This study confirms that the depression, as a mental illness, alters the frontal EEG signals of clinical depression patients. The main results demonstrate that the complexity, evaluated by both sample entropy and LZC, has increased significantly in depression patients compared with healthy group. Furthermore, the complexity escalates as the depression severity deepens. To the best of our knowledge, there were barely any previous studies to evaluate the depression severities by SEn or LZC.

Theoretically, sample entropy and Lempel–Ziv complexity are proposed based on different mathematical algorithm. However, they are both dedicated to evaluating the complexity of physiological signals as nonlinear features. As discussed above, the SEn measures the irregularity of the data that is related to signal complexity [29], while the LZC values the sequence complexity by counting the rate of new patterns appearing in a time series. Therefore, the increasing of SEn and LZC values both suggests increased variability and unpredictability of the investigated series. Interestingly, in literature reading, the authors found that those previous studies, which explored the complexity difference between depressed and healthy people by employing SEn and LZC method separately, presented inconsistent results. Most studies concluded an increasing complexity in depression patients with higher LZC values [5, 14], while the majority of SEn studies speculated decreased complexity with lower SEn values in patients [18, 19]. Furthermore, even by employing the same parameter, different or even opposite results could be obtained; i.e., increased SEn was presented from depression patients by Cukic with even superior performance in depression discrimination compared with Higuchi's fractal dimension method [29]. That is why this study employs both SEn and LZC simultaneously to explore the complexity variation in depression patients.

However, consistent results have been obtained in this study, which is that the EEG complexity has significant increase in depression patients compared with healthy group, confirmed by increased values of both SEn and LZC. The inconsistent results mentioned above might be caused by channels from different brain regions in EEG measurement, different frequency band used in EEG analysis, or even different parameters employed in SEn calculation as it is sensitive to the tolerance threshold *r*. This study focused on the alpha band EEG (8∼13 Hz) collected from poles of left prefrontal lobe Fp1, right prefrontal lobe Fp2, and forehead center Fz. And the accuracy of this study could be confirmed by the consistence to most literatures, as well as conformity between SEn and LZC. Besides, the significantly higher SEn and LZC values from this study confirm the importance of frontal region in depression recognition [14]. Furthermore, it is suggested that the complex pattern of autonomic regulation was affected by the inhibitory function of the frontal cortex on subcortical structure; therefore, the brain activity of frontal cortex is linked to neurocardiac dynamic [15, 30, 31]. In line with this speculation, the increased irregularity and unpredictability of prefrontal lobe activity found in this study could provide interpretation that the depression disturbs brain neurophysiology [5] and the central nervous system and therefore alters heart rate variability and cardiorespiratory coupling of depression patients [23, 32–34].

The article "Frontal Alpha Complexity of Different Severity Depression Patients" was published in 2020. Journal: J Healthc Eng.

Besides, in current depression, timely diagnosis and treatment especially of mild depression are of particularly importance, which could help take precautions previously and avoid further evolution into major depression [35]. However, this is also the challenge for clinical diagnosis as the mild depression patients would reveal less clinical manifestation and even conceal some facts on purpose, which leads to missed diagnosis finally. Fortunately, in this study SEn shows up its superiority in distinguishing mild depression from healthy subjects. As shown in Figure 3, even for the Non-De group which contains patients with no clinical depressive state, SEn values of three channels still all exhibit significantly increases compared with healthy group, with increases of 0.0081 for SEn_Fp1, 0.0079 for SEn_Fz, and 0.0100 for SEn_Fp2. In this respect, SEn performs better than LZC method in mild depression recognition. However, LZC_Fp2 shows comparatively steady increasing among four groups, and LZC measures exhibit better correlation between depression severities and HDRS scores.

Figure 3 presents an overall gradually rising trend of SEn and LZC as the depression deepens with the exception that the three SEn measures and LZC_Fp1 of Con-De group show unexpected decrease compared with Mil-De. This phenomenon might result from pharmacological action, and the Con-De group was under the heaviest drug does. Previous studies found that antidepressant medications with thymoleptic properties generated a decline of alpha activity and induced a slight decline in the prefrontal brain activity [11, 36]. The sudden decrease of Con-De further leads to the negative correlation between SEn values and the HDRS scores in the correlation analysis.

The article "Frontal Alpha Complexity of Different Severity Depression Patients" was published in 2020. Journal: J Healthc Eng.

This study has several limitations. Firstly, the medication and gender factors should be taken into consideration in future experiment design. Besides, this study only focused on frontal alpha band EEG; more EEG bands or even full band EEG from different brain regions could be analyzed in the future to get more complete understanding of depressive brain.

## 5. Conclusions

In summary, this study employed both SEn and LZC to explore the EEG complexity variation among different severity depressions. The results suggest increased frontal alpha complexity in depression patients compared with healthy group, and the increase rises as the depression deepens. This variation of EEG signal provides interpretation of the alteration of depression brain neurophysiology as well as the patients' physiological change. Finally, SEn and LZC are suggested as promising biomarkers in future computer-aided diagnosis of depression, and SEn is especially superior in mild depression recognition.

## Figures and Tables

**Figure 1:** Pole locations of international 10–20 system. Three poles used in this study, Fp1, Fz, and Fp2 were marked in orange.

**Figure 2:** Complexity distribution among different depression severities and healthy controls. Each panel shows one of the six features distribution among four groups: (a)–(c) sample entropy of Fp1, Fz, and Fp2 poles, (d)–(f) Lempel–Ziv complexity of three poles. The mean feature value of each group is shown by the height of the bar, while the standard error shown by the length of the horizontal bar exceeding the main bar. “*∗*”: significant difference with *p* < 0.05. “*∗∗*”: significant difference with *p* < 0.01.

**Figure 3:** Correlation analysis between feature values and HDRS scores. All correlation index *R* and *p* values are given in Table 3, and linear fit line is also given if there is significant correlation. The scatter plots represent complexity values of all subjects.

**Table 1:** Subjects' information.

	Group			
	Depression patients			
	Healthy	Non-De	Mil-De	Con-De
No.	14	15	34	20
Age (years)	45 ± 15	47 ± 16	42 ± 16	44 ± 15
Education, ≤12 years/≥13 years	3/11	13/2	30/4	14/6
Occupation, yes/no	12/2	12/3	22/12	12/8
Right handedness, yes/no	13/1	14/1	34/0	17/3
Smoking, yes/no	3/11	3/12	3/31	3/17
Depression type, MDD/bipolar disorder	—	13/2	31/3	16/4
HDRS score	—	3.93 ± 2.52	13.17 ± 3.00	20.85 ± 2.20

Data are expressed as number or mean ± standard deviation (std).

The article "Frontal Alpha Complexity of Different Severity Depression Patients" was published in 2020. Journal: J Healthc Eng.

**Table 2:** Index values of each group and difference significance results.

	Chi-square	Healthy	Non-De	Mil-De	Con-De
	(Kruskal–Wallis rank test)				
SEn_Fp1	54.07^∗∗^	0.6529 ± 0.0008	0.6610 ± 0.0011^aa^	0.6615 ± 0.0007^aa^	0.6576 ± 0.0009^aabcc^
SEn_Fz	61.67^∗∗^	0.6517 ± 0.0008	0.6596 ± 0.0010^aa^	0.6619 ± 0.0008^aa^	0.6594 ± 0.0009^aa^
SEn_Fp2	80.54^∗∗^	0.6507 ± 0.0008	0.6607 ± 0.0010^aa^	0.6616 ± 0.0007^aa^	0.6583 ± 0.0009^aacc^
LZC_Fp1	41.25^∗∗^	0.9191 ± 0.0014	0.9200 ± 0.0019	0.9290 ± 0.0012^aabb^	0.9276 ± 0.0014^aabb^
LZC_Fz	33.18^∗∗^	0.9217 ± 0.0015	0.9180 ± 0.0019	0.9278 ± 0.0011^aabb^	0.9289 ± 0.0014^aabb^
LZC_Fp2	50.32^∗∗^	0.9181 ± 0.0014	0.9194 ± 0.0020	0.9282 ± 0.0012^aabb^	0.9291 ± 0.0012^aabb^

^1^ Feature values of each group and the results of difference analysis are shown in this table. Feature values are expressed as mean ± standard error (SE). ^∗∗^Statistical difference significance among four groups with *p* < 0.01. ^aa^Significant difference compared with healthy group with *p* < 0.01.^b^Significant difference compared with Non-De group with *p* < 0.05. ^bb^Significant difference compared with Non-De group with *p* < 0.01. ^cc^Significant difference compared with Mil-De group with *p* < 0.01.

**Table 3:** Regression equations between six features and HDRS scores.

Regression equation:	*R*-value	*R* ^2^-value	*p* value
SEn_Fp1 = −0.0003 ^∗∗^ HDRS score + 0.6636^∗∗^	−0.1284	0.0165	0.0009
SEn_Fz = −0.0001 ^∗^ HDRS score + 0.6616	−0.0364	0.0013	0.3484
SEn_Fp2 = −0.0002 ^∗^ HDRS score + 0.6630^∗^	−0.0990	0.0098	0.0107
LZC_Fp1 = 0.0002 ^∗^ HDRS score + 0.9242	0.0548	0.0030	0.1581
LZC_Fz = 0.0003 ^∗^ HDRS score + 0.9214^∗∗^	0.1067	0.0114	0.0059
LZC_Fp2 = 0.0002 ^∗^ HDRS score + 0.9234	0.0735	0.0054	0.0582

^∗∗^Significant correlation with *p* < 0.01.^∗^Significant correlation with *p* < 0.05.

## Data Availability

The datasets for this manuscript are not publicly available because patients' privacy is involved in this study and confidentiality agreement was signed to prevent information leakage. Requests to access the datasets should be directed to Licai Yang (yanglc_sdu@163.com) and Chengyu Liu (chengyu@seu.edu.cn).

## References

[1] WHO (2020). *Depression Availabe Online*.

[2] Zhang F.-F., Peng W., Sweeney J. A., Jia Z.-Y., Gong Q.-Y. (2018). Brain structure alterations in depression: psychoradiological evidence. *CNS Neuroscience & Therapeutics*.

[3] Akdemir Akar S., Kara S., Agambayev S., Bilgiç V. (2015). Nonlinear analysis of EEGs of patients with major depression during different emotional states. *Computers in Biology and Medicine*.

[4] Lanzotti A., Martorelli M., Maietta S., Gerbino S., Penta F., Gloria A. (2019). A comparison between mechanical properties of specimens 3D printed with virgin and recycled PLA. *Procedia CIRP*.

The article "Frontal Alpha Complexity of Different Severity Depression Patients" was published in 2020. Journal: J Healthc Eng.

[5] Bachmann M., Päeske L., Kalev K. (2018). Methods for classifying depression in single channel EEG using linear and nonlinear signal analysis. *Computer Methods and Programs in Biomedicine*.

[6] Cai H., Han J., Chen Y. (2018). A pervasive approach to EEG-based depression detection. *Complexity*.

[7] Grin-Yatsenko V. A., Baas I., Ponomarev V. A., Kropotov J. D. (2010). Independent component approach to the analysis of EEG recordings at early stages of depressive disorders. *Clinical Neurophysiology*.

[8] Dan V. I., Greenwald S., Devlin P. (2009). Frontal EEG predictors of treatment outcome in major depressive disorder. *European Neuropsychopharmacology*.

[9] Salustri C., Tecchio F., Zappasodi F. (2007). Cortical excitability and rest activity properties in patients with depression. *Journal of Psychiatry &amp; Neuroscience: JPN*.

[10] Hosseinifard B., Moradi M. H., Rostami R. (2013). Classifying depression patients and normal subjects using machine learning techniques and nonlinear features from EEG signal. *Computer Methods and Programs in Biomedicine*.

[11] Acharya U. R., Sudarshan V. K., Adeli H., Santhosh J., Koh J. E. W., Adeli A. (2015). Computer-aided diagnosis of depression using EEG signals. *European Neurology*.

[12] Malloy P. F., Cohen R. A., Jenkins M. A., Paul R. H. (2006). *Frontal Lobe Function and Dysfunction*.

[13] Paul W., Burgess I. H. R. (2002). *Principles of Frontal Lobe Function*.

[14] Kalev K., Bachmann M., Orgo L., Lass J., Hinrikus H. Lempel-Ziv and multiscale Lempel-Ziv complexity in depression.

[15] Chang J. S., Yoo C. S., Yi S. H. (2012). An integrative assessment of the psychophysiologic alterations in young women with recurrent major depressive disorder. *Psychosomatic Medicine*.

[16] Lee P. F., Kan D. P. X., Croarkin P., Phang C. K., Doruk D. (2018). Neurophysiological correlates of depressive symptoms in young adults: a quantitative EEG study. *Journal of Clinical Neuroscience*.

[17] Richman J. S., Moorman J. R. (2000). Physiological time-series analysis using approximate entropy and sample entropy. *American Journal of Physiology Heart & Circulatory Physiology*.

[18] Faust O., Ang P. C. A., Puthankattil S. D., Joseph P. K. (2014). Depression diagnosis support system based on eeg signal entropies. *Journal of Mechanics in Medicine and Biology*.

[19] Acharya U. R., Sudarshan V. K., Adeli H. (2015). A novel depression diagnosis index using nonlinear features in EEG signals. *European Neurology*.

[20] Bruder G. E., Stewart J. W., McGrath P. J. (2017). Right brain, left brain in depressive disorders: clinical and theoretical implications of behavioral, electrophysiological and neuroimaging findings. *Neuroscience & Biobehavioral Reviews*.

The article "Frontal Alpha Complexity of Different Severity Depression Patients" was published in 2020. Journal: J Healthc Eng.

[21] Ferenets R., Lipping T., Anier A., Jantti V., Melto S., Hovilehto S. (2006). Comparison of entropy and complexity measures for the assessment of depth of sedation. *IEEE Transactions on Biomedical Engineering*.

[22] Zhang Z. (2005). Emotion evaluation. *Behavioral Medicine Scale Manual*.

[23] Zhao L., Yang L., Su Z., Liu C. (2019). Cardiorespiratory coupling analysis based on entropy and cross-entropy in distinguishing different depression stages. *Frontiers in Physiology*.

[24] Liu C., Zhang C., Zhang L., Zhao L., Liu C., Wang H. (2015). Measuring synchronization in coupled simulation and coupled cardiovascular time series: a comparison of different cross entropy measures. *Biomedical Signal Processing and Control*.

[25] Zhao L., Wei S., Zhang C. (2015). Determination of sample entropy and fuzzy measure entropy parameters for distinguishing congestive heart failure from normal sinus rhythm subjects. *Entropy*.

[26] Lempel A., Ziv J. (1976). On the complexity of finite sequences. *IEEE Transactions on Information Theory*.

[27] Li Y., Tong S., Liu D. (2008). Abnormal EEG complexity in patients with schizophrenia and depression. *Clinical Neurophysiology*.

[28] Kaspar F., Schuster H. G. (1987). Easily calculable measure for the complexity of spatiotemporal patterns. *Physical Review A*.

[29] Cukic M., Pokrajac D., Stokic M., Simic S., Radivojevic V., Ljubisavljevic M. (2018). EEG machine learning with Higuchi fractal dimension and Sample Entropy as features for successful detection of depression. https://arxiv.org/abs/1803.05985.

[30] Ziegler G., Dahnke R., Yeragani V. K., Bär K.-J. (2009). The relation of ventromedial prefrontal cortex activity and heart rate fluctuations at rest. *European Journal of Neuroscience*.

[31] Chang J. S., Yoo C. S., Yi S. H. (2010). Changes in heart rate dynamics of patients with schizophrenia treated with risperidone. *Progress in Neuro-Psychopharmacology and Biological Psychiatry*.

[32] Chen X., Yang R., Kuang D. (2017). Heart rate variability in patients with major depression disorder during a clinical autonomic test. *Psychiatry Research*.

[33] Paniccia M., Paniccia D., Thomas S., Taha T., Reed N. (2017). Clinical and non-clinical depression and anxiety in young people: a scoping review on heart rate variability. *Autonomic Neuroscience*.

[34] Yeh T.-C., Kao L.-C., Tzeng N.-S. (2016). Heart rate variability in major depressive disorder and after antidepressant treatment with agomelatine and paroxetine: findings from the Taiwan Study of Depression and Anxiety (TAISDA). *Progress in Neuro-Psychopharmacology and Biological Psychiatry*.

The article "Frontal Alpha Complexity of Different Severity Depression Patients" was published in 2020. Journal: J Healthc Eng.

[35] Li X., La R., Wang Y. (2019). EEG-based mild depression recognition using convolutional neural network. *Medical & Biological Engineering & Computing*.

[36] Hunter A. M., Leuchter A. F., Morgan M. L., Cook I. A. (2006). Changes in brain function (quantitative EEG cordance) during placebo lead-in and treatment outcomes in clinical trials for major depression. *American Journal of Psychiatry*.

